This article has been retracted.

# Association of *β*2-Agonist Receptor Gene Polymorphisms with Acute Exacerbations of COPD: A Prospective Observational Study

**DOI:** 10.1155/2022/2711489

**Published:** 2022-09-12

**Authors:** Fengfeng Lu, Nengluan Xu, Jianshi Zheng

**Affiliations:** Department of Pulmonary and Critical Care Medicine, Fujian Provincial Hospital, Fuzhou 350000, China

## Abstract

**Objective:**

To investigate the relationship between *β*2-agonist receptor gene polymorphisms and acute exacerbations of chronic obstructive pulmonary disease (COPD).

**Methods:**

Retrospective analysis of 99 patients in the respiratory and critical care unit of Fujian Provincial Hospital from 2018 to 2020. The clinical characteristics of different genotypes were compared, and the treatments of different genotypes and the analysis of factors associated with acute exacerbations of COPD were compared.

**Results:**

During the 12-month follow-up period, 53 patients developed acute exacerbations, with the 16Arg/Arg homozygous requiring significantly more antibiotics and hormones than the other two genotypes; when agonist receptor 16 gene polymorphism was associated with the risk of acute exacerbation, 16Arg/Gly patients had a 5.286-fold increased risk of acute exacerbation (OR = 6.286, 95% CI. 1.476–26.759, *P*=0.013). 16Arg/Arg patients had a 5.060-fold increased risk of acute exacerbation (OR = 6.060, 95% confidence interval: 1.407–26.161, *P*=0.016).

**Conclusion:**

Acute exacerbation of 16Arg/Arg COPD is very serious; 16Arg/Gly increases the risk of acute exacerbation in COPD patients; and provides help for future treatment and management options of the disease.

## 1. Introduction

Chronic obstructive pulmonary disease (COPD) is one of the most common chronic diseases of the respiratory system and is a global public health problem [1]. Chronic obstructive pulmonary disease (COPD) is a dynamic chronic disease characterized by persistent respiratory symptoms and or airflow limitation, which can be prevented and treated [2]. In China, the prevalence of COPD in people over 40 years of age is 13.7% [3] and is expected to be the 3rd leading cause of death worldwide by 2020 [4]. Acute exacerbation of chronic obstructive pulmonary disease (AECOPD) is an acute worsening of a patient's existing respiratory symptoms (mainly manifested as worsening dyspnea and increased cough and sputum) beyond the patient's daily variation and causes the patient to require additional medication [5]. Acute exacerbations account for 70% of the disease in clinical practice, so it is generally accepted that acute exacerbations of COPD are key events in the development and progression of the disease, and are important indicators for assessing patients' future health status and disease prognosis [6]. The total annual per capita cost accounts for 40% of the average total household income in China in that year (for urban patients associated with COPD), and the economic burden is more severe in rural areas [7]. Patients with COPD experience 0.5–3.5 acute exacerbations per year, with some COPD patients having at least 2 acute exacerbations per year, which we usually define as frequent acute exacerbations [8]. Patients with frequent exacerbations have higher morbidity and mortality, poorer health status, and more severe economic impact than patients with infrequent exacerbations [9, 10]. In recent years, there has been increasing interest in the role of genetic factors in the pathogenesis and pharmacological efficacy of COPD.

Inhaled *β*-agonists are one of the main bronchodilators in the treatment of COPD [11]. *β*2-adrenergic receptor (ADRB2) is a G protein-coupled transmembrane receptor that is highly expressed in lung tissue, and activation of this receptor has the function of relaxing bronchial smooth muscle, anti-inflammatory and improving airway epithelial mucus [12]. adrB2 is located on chromosome 5q31–32. It is an intronless, relatively small gene encoding 413 amino acids [13]. At least five single nucleotide polymorphisms (SNPs) have been identified so far, namely, +46A/G, 79C/G, +100G/A, +491C/T, and −47C/T, corresponding to nucleotide variant sites 16, 27, 34, 164, and 19. Most of the existing studies have focused on 16 [16Arg > Gly; rs 1042713] and 27 [27Gln > Glu; rs 1042714] variants.

Previous high-quality studies examining the clinical characteristics of patients with frequent acute exacerbations of COPD are not numerous, and some of the findings are still inconsistent. Studies [14] have shown that typing of chronic obstructive pulmonary disease (COPD) is an independent predictor to assess the frequency of their future acute exacerbations. In recent years, literature and foreign guidelines have pointed out that better outcomes have been obtained with targeted and individualized treatment after the phenotypic classification of COPD [15]. It is suggested that different COPD phenotypes have different characteristics, and more valuable findings may be obtained if the clinical characteristics of patients with frequent acute exacerbations (FE) of COPD are sought on the basis of phenotypes. The aim of this study is to analyze the clinical characteristics of different COPD patients, to find the possible risk factors for each COPD frequent acute exacerbation (FE), and to compare and generalize them, which can eventually provide targeted individualized treatment for patients, reduce the frequency of future acute exacerbations, and promote the development of precision medicine.

## 2. Research Methodology

### 2.1. Patient Data

Ninety-nine patients from the Department of Respiratory and Critical Care Medicine of Fujian Provincial Hospital from 2018 to 2020 were included in this study.

#### 2.1.1. Inclusion Criteria

1. Meet the diagnostic criteria for acute exacerbation of chronic obstructive pulmonary disease [16]. Acute deterioration of the patient's original respiratory symptoms (mainly manifested by increased dyspnea and cough and sputum) beyond the patient's daily variation and leading to the patient's need for additional medication.
2. Patients aged 40–85 years.

#### 2.1.2. Exclusion Criteria

1. Combination of other serious lung diseases, such as active tuberculosis, lung cancer, diffuse interstitial pulmonary fibrosis, and bronchiectasis
2. Combination of cardiovascular, cerebrovascular, hepatic and renal, hematopoietic systems and other serious primary diseases, psychiatric patients, such as cerebral hemorrhage and massive cerebral infarction, chronic cardiac insufficiency, acute myocardial infarction, uremia, lymphoma, and leukemia
3. Recent use of immunosuppressive drugs, long-term glucocorticoid therapy, and the presence of serious immune system diseases

### 2.2. Clinical Information

Clinical data including demographic data, smoking status, blood gas analysis, baseline lung function, and bronchial dilation test results were obtained through the electronic medical record system. A questionnaire was used for all patients to obtain the number of hospitalizations due to acute exacerbations, systemic glucocorticoid use, and antibiotic use in the past 12 months. At the same time, venous blood samples were collected from each patient for ADRB2 gene polymorphism detection.

### 2.3. Gene Polymorphism Detection Process

DNA extraction kit (Guangzhou Meiji Bio, HiPure Universal DNA Kit) was used for DNA extraction, and gene amplification was performed on a Bio-rad T-100 PCR instrument. Primers: upstream: ACATAACGGGCAGAACGCAC, downstream: CGATGAGAGACATGACGATGC, select qualified PCR products were genotyped by next-generation sequencing on an ABI 3730 sequencer.

### 2.4. Statistical Methods

SPSS 17.0 software was used for analysis. Measurement data were expressed as mean ± standard deviation ($\bar{x}\pm s$), and differences between groups were analyzed by variance analysis; count data were expressed as rates, and differences between groups were analyzed by chi-square test. Binary Logistic was used to analyze the association between gene polymorphisms and acute exacerbation. Two-sided *P* < 0.05 was considered statistically significant.

## 3. Statistical Results

### 3.1. Clinical Features

A total of 99 patients with the chronic obstructive pulmonary disease were included in this analysis, with an average age of (69.38 ± 6.69) years, (52–83) years old, 96 males, 20 Arg/Arg, 61 Arg/Gly, and 18 Gly/Gly. There was no significant difference in the smoking index, FEV1, FEV1% and FEV1/FVC, CAT score, mMRC, number of acute exacerbations, and drug combination (all *P* > 0.05). The difference between the types was statistically significant (*P* < 0.05, Tables 1 and 2). Furthermore, binary logistic regression analysis showed that the risk of acute exacerbation increased by 5.286 times (OR = 6.286, 95% CI: 1.476∼26.759, *P*=0.013) in the heterozygous genotype Arg/Gly, and still increased by 5.060 times after adjusting for FEV1 OR = 6.060, 95% CI: 1.407∼26.161, *P*=0.016, Table 3).

## 4. Discussion

Chronic obstructive pulmonary disease (COPD) is a common disease typically characterized by incomplete reversible airflow limitation and persistent respiratory symptoms. As the disease progresses, lung function declines progressively, leading to a reduced workforce and, in severe cases, respiratory failure, pulmonary heart disease, and even death. According to the results of a recent large epidemiological cross-sectional survey in China, the prevalence of COPD defined by spirometry reached 8.6%, and there are nearly 100 million COPD patients nationwide, second only to hypertension and diabetes, and this data is on the rise, which urgently needs the attention of the whole society [17]. The active search for clinical factors or biomarkers that predict the future risk of frequent acute exacerbations in COPD patients is an important clinical event at present.

It was found [18] that among the 16 focal polymorphisms of the ADRB2 gene, those carrying the Arg/Arg isoform required antibiotics and systemic hormones in the event of an acute exacerbation, indicating a more severe condition; those with the 16Arg/Gly isoform had a higher risk of acute exacerbation. Studies [19,20] found that 16Arg/Gly and 27Gln/Glu polymorphisms by themselves did not affect airflow limitation. Our study found no significant differences in pulmonary function indicators between ADRB2 genotypes, but they may lead to an increased risk of exacerbations, as well as to different severity of the disease. Currently, only a few studies have analyzed the role of ADRB2 gene polymorphisms in COPD and the application of antibiotics and systemic hormones. The study [21] found a significant increase in the use of antibiotics and hormones in patients with 16Arg/Arg COPD during acute exacerbations, but did not affect the number of hospitalizations associated with acute exacerbations consistent with the results of this study. Similarly, the study [22] found no relationship between ADRB2 polymorphism and the number of hospitalizations associated with COPD exacerbations. At present, the mechanism by which ADRB2 gene polymorphisms are associated with the severity of COPD exacerbations remains unclear. According to Ligert's theory, ADRB2 containing the glycine 16 position may be downregulated by exposure to endogenous catecholamines [23]. All of the patients we included had severe to very severe COPD. Most of the patients were treated with beta-agonists and the receptors were more significantly downregulated. As a result, they were more prone to respiratory infections and required more hormones.

Most of the current studies on the association of ADRB2 gene polymorphisms with exacerbations of COPD are on the risk of acute exacerbations when inhaling *β*-agonists with different genotypes [24]. In a subgroup analysis of the POET-COPD trial, patients inhaling salmeterol with genotype Arg/Arg had a significantly lower risk of acute exacerbations than Arg/Gly and Gly/Gly, although we did not specifically include patients who received beta-agonists. These patients were treated with *β*-agonists, but they all received *β*-agonists because of the severity of their disease. Therefore, it can be stated that the above findings are consistent with ours. However, in other clinical trials, the ADRB2 gene polymorphism was not associated with acute exacerbations in COPD patients who inhaled long-acting beta-agonists. Therefore, the study [25] was systematically reviewed after including all the above-mentioned trials and found no statistical differences.

The relationship between ADRB2 gene polymorphisms and acute exacerbations of inhaled beta-agonists in COPD patients remains unclear. The study [26] found that airway smooth muscle cells expressing the Arg allele had less receptor downregulation when exposed to *β*-receptor agonists compared to airway smooth muscle cells expressing the Gly allele in an in vitro study.

## 5. Conclusion

Patients with different phenotypes of frequent acute exacerbations (FE) of chronic obstructive pulmonary disease (COPD) may have their own distinct clinical manifestations. Our study found that 16Arg/Arg COPD worsens severely; 16Arg/Gly increases the risk of acute exacerbations in COPD patients, which may help identify risk factors for COPD that are more likely to lead to increased frequency of hospitalization, and provide assistance for future disease diagnosis and management programs.

## Figures and Tables

**Table 1:** Comparison of clinical characteristics of different genotypes.

	Arg/Arg (*n* = 20)	Arg/Gly (*n* = 61)	Gly/Gly (*n* = 18)	F value/chi-square	*P* value
Age	70.60 ± 7.05	69.33 ± 6.52	68.22 ± 7.01	0.599	0.551
Male	20	58	18	1.927	0.382
Smoking index	49.68 ± 31.92	46.07 ± 30.28	45.69 ± 30.56	0.117	0.890
FEV1 (L)	0.84 ± 0.22	0.93 ± 0.31	0.97 ± 0.27	1.203	0.305
FEV1 (%)	32.71 ± 8.94	36.86 ± 11.86	36.02 ± 9.91	1.072	0.346
FEV1/FVC (%)	38.58 ± 10.72	39.12 ± 10.26	44.35 ± 9.08	2.070	0.132
CATscore	15.30 ± 4.89	15.23 ± 6.45	14.44 ± 6.30	0.127	0.881
mMRC	2.45 ± 1.00	2.25 ± 1.06	1.72 ± 1.13	2.439	0.093
Exacerbations	16 (80.0%)	30 (49.2%)	7 (38.9%)	7.649	0.022

*Note.* FEV1, FVC, CAT, mMRC.

**Table 2:** Comparison of treatment methods for different genotypes.

	Arg/Arg	Arg/Gly	Gly/Gly		
LAMA	0	5 (8.2%)	1 (5.6%)	1.511	0.825
LABA + ICS	1 (5.0%)	9 (14.8%)	3 (16.7%)		
ICS + LABA + LAMA	19 (95.0%)	47 (77.0%)	14 (77.8%)		
*Antibiotics used*					
0	8 (40.0%)	31 (50.8%)	12 (66.7%)	14.944	0.021
1	2 (10.0%)	17 (27.9%)	6 (33.3%)		
2	6 (30.0%)	6 (9.8%)	0		
≥3	4 (20.0%)	7 (11.5%)	0		
*Number of hormones*					
0	13 (65.0%)	40 (65.6%)	14 (77.8%)	14.732	0.022
1	1 (5.0%)	17 (27.9%)	4 (22.2%)		
2	4 (20.0%)	2 (3.3%)	0		
≥3	2 (10.0%)	2 (3.3%)	0		
*Number of acute exacerbations*					
0	5 (25.0%)	31 (50.8%)	11 (61.1%)	12.558	0.051
1	6 (30.0%)	12 (19.7%)	7 (38.9%)		
2	5 (25.0%)	10 (16.4%)	0		
≥3	4 (20.0%)	8 (13.1%)	0		

*Note.* LAMA, LABA, LAMA.

**Table 3:** Correlation between rs 1042713 and acute exacerbation of the chronic obstructive pulmonary disease.

	B	S.E,	Wals	*P*	Exp (B)	95% of EXP (B) C.I.	
						Lower limit	Higher limit
Arg/Arg			6.864	0.032	Ref		
Arg/Gly	1.838	0.739	6.186	0.013	6.286	1.476	26.759
Gly/Gly	0.419	0.547	0.587	0.444	1.521	0.520	4.444
Arg/Arg^1^			6.498	0.039	Ref		
Arg/Gly	1.802	0.745	5.848	0.016	6.060	1.407	26.101
Gly/Gly	0.408	0.548	0.553	0.457	1.504	0.513	4.404

*Note.* ^1^Adjustment factor is FEV1.

## Data Availability

The simulation experiment data used to support the findings of this study are available from the corresponding author upon request.
